# Correlation between Endoscopic Morphology and Bleeding of Gastric Ulcer

**DOI:** 10.1155/2022/2169551

**Published:** 2022-02-24

**Authors:** He Xiaohua

**Affiliations:** Department of Emergency, Ganzhou People's Hospital, Ganzhou, Jiangxi 341000, China

## Abstract

**Objective:**

To improve the safety and reliability of gastric ulcer treatment, the emergence of digestive endoscopy technology in recent years has become a conventional method for the diagnosis of peptic ulcer bleeding. Endoscopic characteristics can judge the severity of patients more accurately and comprehensively, provide a basis for follow-up treatment, and judge the prognosis.

**Methods:**

298 patients with a suspected gastric ulcer who underwent laryngeal gastroduodenal endoscopy and confirmed gastroduodenal ulcer in our hospital in recent half a year were randomly selected. Olympus cv-170 electronic gastroscope machine was used to carry out gastroscopy for patients with gastric ulcers, analyze, and judge the number of bleeding cases in different stages of treatment, such as lesion type, lesion location, patient age, and gender. The statistics of bleeding cycle and bleeding volume, prognosis recovery, and the correlation of different risk levels were analyzed.

**Results:**

After examination and diagnosis, the patients were followed up for one year. According to the number of bleeding cases, bleeding cycle, and bleeding volume of patients with different ulcer locations in the acute stage, healing stage, and scar stage, the distribution of bleeding cases of different ulcer locations in different stages was roughly the same, and there was no significant difference. The proportion of bleeding cases in the acute stage was the highest, while the proportion in the healing stage was the lowest. The number of bleeding cases, bleeding cycle, bleeding volume, and related symptoms in patients with gastric ulcers during the treatment were significantly correlated with those in the acute stage, healing stage, and scar stage. There was no significant difference in the distribution of bleeding in one year among different stages of ulcer in the same age group, however, the bleeding in one year would be more serious with the increase of age in different age groups. Gender differences have a great impact on the bleeding of the ulcer within one year. It usually shows that the bleeding of ulcers in males is more serious than that in females.

**Conclusion:**

The location and pathological development of gastric ulcers can be found in time through gastroscopy, and the status of gastroscopy can be analyzed. Most gastric ulcers are acute bleeding. The amount of bleeding has little correlation with the stage of gastric ulcer, and it is related to the location of bleeding. The older the age, the greater the amount of bleeding, and the amount of bleeding in men is greater than that in women. In the treatment of gastric ulcers, gastroscopy, as a doctor's examination and treatment method, effectively improves the safety and reliability of clinical treatment of gastric ulcer bleeding and reduces the adverse risk.

## 1. Instruction

Gastric ulcer is a common chronic disease of the digestive system. It is caused by the damage of gastric mucosa exceeding the mucosal muscle layer. Most of the parts of the disease are the esophagus, stomach, or duodenum. Duodenal ulcer is also known as peptic gastric ulcer. Gastric ulcer disease will have varying degrees of pain in the abdomen, which is easy to cause gastric bleeding, gastric perforation, and other complications. It brings great harm to the patient's body. Gastric ulcer bleeding is a common clinical disease with the characteristics of high prevalence and long course of disease. When it is serious, it will lead to complications, such as heart and cerebral infarction. The initial symptoms of gastric ulcer are not obvious. The common symptoms are gastric distention, stomachache, poor appetite, nausea, and acid reflux. Most people do not pay much attention to it, which leads to the disease if not treated in time. In severe cases, it will be accompanied by gastric bleeding.

At present, endoscopy is the first choice for the diagnosis of gastric ulcer. It can not only diagnose the location, size, shape, inflammation of surrounding mucosa and other diseases but also can biopsy the lesions under direct vision.

As the preferred method for routine detection of the stomach, endoscopy provides a basis for doctors to judge the pathology of patients with the help of gastric ulcer and bleeding. They can be seen by endoscopy doctors, and they formulate the best treatment plan based on this judgment to improve the treatment effect.

After treatment, although the basal surface of the ulcer is clean, there is still some erosion around the ulcer and bleeding. In severe cases, it can lead to massive bleeding and affect the prognosis. At present, the classification of gastric ulcer does not pay attention to the influence of gastroscopic characteristics of mucosal erosion around ulcer on bleeding. This study makes statistics on the gastroscopic characteristics of ulcer itself and its surrounding mucosal erosion and analyzes its bleeding status and the correlation of different risk levels to help better judge the bleeding and prognosis of patients.

By analyzing the bleeding status of a gastric ulcer, this study discussed gastroscopy as an effective clinical method for the treatment of peptic ulcer bleeding, provided a safer and effective basis for the clinical treatment of peptic ulcer bleeding, and played a positive role in the treatment scheme of gastric ulcer.

## 2. Literature Review

Xie Wenli: to explore the clinical effect of digestive endoscopy combined with quadruple therapy in gastric ulcer, this paper uses the reference group for comparison and comes to the conclusion that the combined application of digestive endoscopy and quadruple therapy can improve the curative effect of gastric ulcer [1]. Han Peng: to explore the compliance of clinical nursing during endoscopic examination of elderly gastric ulcer, the reference group is used for comparison, and it is concluded that the implementation of clinical nursing during endoscopic examination of elderly gastric ulcer patients can improve the compliance of examination to reduce the occurrence of adverse reactions [2]. Pan Qilong: to study the effect of esomeprazole combined with Kangfuxin solution on ulcer mucosal healing of gastric ulcer bleeding, esomeprazole alone and esomeprazole combined with Kangfuxin solution were compared in this paper [3]. The results show that the effect of esomeprazole combined with Kangfuxin solution is higher than that of esomeprazole alone, which can improve the patients' quality of life. The blood effect is related to the quality of ulcer mucosal healing, and it does not increase the risk of adverse effects. Wang Fengxia discussed the influencing factors of gastric bleeding in patients with gastric ulcer [4]. Wang Xiang (2021): through the combination of Chinese and Western medicine in the treatment of gastric ulcer, to explore the therapeutic effect of Xiangsha Yangwei pill and Rabeprazole on gastric ulcer and TGF in gastric mucosa-*β*_ 1 expression, it is concluded that the combination of Chinese and Western medicine improves the therapeutic effect of gastric ulcer [5]. Yuan Xinge's paper discusses the correlation between ultrasonic endoscopy and coagulation indexes in the diagnosis and pathological examination of senile gastric ulcer [6]. Lin Huodong (2021) demonstrated the therapeutic effect of digestive endoscopy combined with quadruple therapy on gastric ulcer bleeding. Through the experimental comparison between the combined group and the quadruple group, it was concluded that digestive endoscopy combined with quadruple therapy can improve the recovery speed of gastric function in patients with gastric ulcer bleeding, eliminate *Helicobacter pylori,* and reduce the incidence of rebleeding [7]. Zhou Shourong demonstrated the therapeutic effect of gastroendoscopy combined with anti-*Helicobacter pylori* quadruple therapy on gastric ulcer bleeding. Through the comparison of the reference group, it was concluded that the treatment of gastroendoscopy combined with anti-*Helicobacter pylori* quadruple therapy for patients with gastric ulcer bleeding can help to eliminate *Helicobacter pylori*, reduce bleeding symptoms, reduce rebleeding rate, and adverse reaction risk [8]. Dai Jing said while studying the influence on patients with gastric ulcer and gastric bleeding that the treatment effect of patients with gastric ulcer and gastric bleeding after intervention is better, which can effectively improve the diet level and medication compliance of patients with gastric ulcer and gastric bleeding and improve the treatment satisfaction of patients with gastric ulcer [9].

## 3. Data and Methods

### 3.1. General Information

298 patients (172 males and 126 females, aged 22 to 58 years, with an average age of 31.5 ± 4.3 years) with suspected gastric ulcer confirmed by laryngogastroduodenal endoscopy in our hospital from January 2020 to June 2020, including 156 cases in the acute stage (95 males and 61 females, aged 23 to 55 years, with an average age of 32.7 ± 4.1 years) and 72 cases in healing stage (44 males and 28 females. The age ranged from 22 to 51 years, with an average age of 30.4 ± 3.8 years). There were 70 cases of scar stage (33 males and 37 females, with an average age of 35.2 ± 4.5 years). According to the location of ulcer, there were 28 cases of the cardia, 35 cases of the gastric bottom, 56 cases of the greater curvature of the stomach, 31 cases of the lesser curvature of the stomach, 75 cases of the antrum and angular notch, 43 cases of the pylorus, and 73 cases of the duodenum.

### 3.2. Inspection Method

Olympus cv-170 electronic gastroscope machine was used for gastroscopy. Lidocaine glue (sulton, ws-209 (x-179)-93) was used for local anesthesia, dimethylsilicone oil emulsion (Percy, 8050-81-5) was used for lubrication and defoaming, and rabeprazole sodium enteric-coated capsule was used for gastric emptying preparation (Jichuan, h20061220). Other drugs, such as lesion staining and microinjury repair, are issued by outpatient doctors based on evidence. During gastroscopy, determine the type and location of lesions. After diagnosis, observe the incidence of gastric bleeding within one year according to the electronic medical record big data system (with the written authorization of the patient before observation), and compare the bleeding time, bleeding volume, bleeding location, and other information.

### 3.3. Statistical Methods

Statistical methods were used to analyze the gastric ulcer, endoscopic morphology, and the bleeding of gastric ulcer. The statistical formulas of mean value and standard deviation rate are as follows:

(1) $$\begin{array}{c} \sigma =\frac{1}{n-1}\sqrt{\overset{n}{\underset{i=1}{\sum }}{\left(x_{i}-\bar{x}\right)}^{2}},\\ \bar{x}=\frac{1}{n}\overset{n}{\underset{i=1}{\sum }}x_{i}, \end{array}$$

*σ*  is the standard deviation rate of input sequence *x*; *x*_*i*_ is the *i* input item in the input sequence *x*; *μ* is the arithmetic mean of the input sequence *x*; *n* is the number of statistical samples.

The *t* value and *P* value of bivariate t-check come from the bivariate t-check process, where *t* value is the value of the output result. When *t* > 10.000, it is considered that there is statistical consistency between the two columns of data, and the greater the *t* value, the greater the consistency. *P* value is the log value of the output result. When *P* < 0.05, it is considered that the result data is within the confidence space. When *P* < 0.01, it is considered that the result data has significant statistical significance. The smaller the *P* value, the higher the degree of confidence. Subject to the length, only the calculation algorithm of *t* value (value) is explained here, as seen in formula (2).

(2) $$\begin{array}{c} t=\frac{\bar{X_{1}}-\bar{X_{2}}}{\sqrt{\left(n_{1}-1\right)\sigma_{1}^{2}+\left(n_{2}-1\right)\sigma_{2}^{2}/n_{1}+n_{2}-2\left(1/n_{1}+1/n_{2}\right)}}. \end{array}$$

$\bar{x}$ is the arithmetic mean of the investigated sample sequence, *μ* is the average value of the reference sample sequence, n is the number of nodes of the investigated sample sequence, m is the number of nodes in the reference sample sequence, and *σ*_*x*_ is the standard deviation rate of the investigated sample sequence.

The *R*^2^ value is obtained by linear regression method under SPSS, and the *t* value and *P* value are obtained by bivariate *t* check. The statistical method of the *R*^2^ value is the ratio of regression residual to mean residual, as shown in formula (3).

(3) $$\begin{array}{c} R^{2}=\frac{\sum {\left(\hat{x}-\bar{x}\right)}^{2}}{\sum {\left(x-\bar{x}\right)}^{2}}. \end{array}$$

$\bar{x}$ is the arithmetic mean of the investigated sample sequence, ${\tilde{x}}_{i}$ is the *i* regression value in the sequence, *x*_*i*_ is the *i* input value in the sequence, and *n* is the number of investigation samples.

## 4. Results

### 4.1. Correlation Analysis of Stage and Location of Gastroduodenal Ulcer on Gastric Bleeding within One Year

Gastroduodenal ulcer is a chronic ulcer that mostly occurs in the stomach. At present, pathology believes that its occurrence is closely related to the action of gastric acid and pepsin. Gastric mucosal erosion is only the inflammation on the surface. During ulcer, the lesion invades the mucosal muscle more deeply. Even if the scar is bound to form with the formation of fibers after healing, the lesion does not involve the muscle layer during erosion, and there is no fiber formation after healing. Hence, there is no scar.

The location of gastroduodenal ulcer is closely related to its bleeding site. In this paper, the positions of the cardia, bottom, great bend, sinus, angular notch, pylorus, and duodenum were taken for endoscopy, as well as the follow-up one-year treatment and clinical observation of bleeding as shown in Table 1.

In Table 1, it can be seen that different stages have little effect on ulcers in different locations. The bleeding proportion in the acute phase is the highest in the same location, and the location of the ulcer plays a decisive role in the amount of bleeding.

In Figure 1, it can be seen that the distribution of bleeding cases in different stages of ulcers at different locations is roughly the same, and there is no obvious difference. They all show that the proportion of bleeding cases in the acute stage is the highest, while the proportion in the healing stage is the lowest.

In Figure 2, it can be seen that ulcers at different locations also have roughly the same distribution in bleeding cycles at different stages. The difference is that the longest bleeding cycle is the healing period, while the shortest bleeding cycle is in the acute period.

In Figure 3, it can be seen that the bleeding volume of ulcers at different positions varies greatly. The bleeding volume of ulcers at the duodenal position is the highest, and the bleeding volume of ulcers at the bottom is the lowest. There was no significant differences in the amount of bleeding in different stages of ulcer.

In Tables 2 and 3, the number of bleeding cases, bleeding cycle, bleeding volume, and related symptoms in patients with gastric ulcer during treatment are significantly correlated with patients in the acute stage, healing stage, and scar stage when the bivariate *t*-test correlation of analysis stage observation data is compared with the nonlinear curve estimation determination coefficient *R*^2^ of analysis observation data.

In Tables 4 and 5, the bivariate *t*-test correlation of the ulcer location observation data and the nonlinear curve estimation determination coefficient R^2^ test correlation of the ulcer location observation data are analyzed and discussed. The comparison results show that the bivariate *T* and the determination coefficient R^2^ test of the specific gastric ulcer location analysis data of the patients are significantly correlated.

### 4.2. Correlation Analysis of Patients' Age and Gender on Gastric Bleeding within One Year

This study followed the patients for a one-year period after examining the diagnosis. Clinical observation was compared with the bleeding cycle and bleeding volume at different ages during different pathology periods. The results are shown in Table 6.

To more intuitively compare the bleeding cycle and bleeding volume of different ages during different pathology periods, visualize the data in the table, and get Figure 4.

In Figure 4, there is no significant difference in the distribution of bleeding in one year among different stages of ulcer in the same age group, however, the bleeding in one year will become more serious with the increase of age in different age groups.

This study followed up the patients for a one-year period after examining the diagnosis. Compare the bleeding cycle and bleeding volume of different sexes. The results are shown in Table 7.

To more intuitively compare the bleeding cycle and bleeding volume of different sexes during different pathology periods, visualize the data in the table, and get Figure 5.

In Figure 5, gender differences have a great impact on the bleeding of ulcers within one year. It usually shows that the bleeding of men is more serious than that of women.

## 5. Discussion

Peptic ulcer often occurs as a chronic ulcer of the stomach and the duodenum. It is a chronic disease with a high incidence rate, which brings suffering to the patient's body. Bleeding is a common form of gastric ulcer. *Helicobacter pylori* infection, gastric ulcer stage A1, gastric ulcer history, smoking history, drinking history, and nonsteroidal anti-inflammatory drugs can affect ulcer bleeding. Daily life maintenance and correct medication are very important.

There are many clinical ways to treat gastric ulcer, most of which are conservative treatment methods. However, the course of treatment is long and the effect is slow. As a new examination method, gastroscopy can quickly judge the bleeding position and gastric condition through gastroscopy, which provides a basis for doctors to issue a treatment plan to achieve the purpose of hemostasis and treatment effect. The gastric ulcer can heal after treatment, however, the severity of the gastric ulcer will affect the recovery process. Therefore, more attention should be paid to the treatment process. Diet and nursing methods need to cooperate with each other to completely improve the situation of the gastric ulcer.

Through the relevant data obtained from this study, gastroscopy effectively improves the safety and reliability of clinical treatment of gastric ulcer bleeding and reduces the adverse risk.

## Figures and Tables

**Figure 1:** Comparison of bleeding cases in different ulcer locations and stages.

**Figure 2:** Comparison of bleeding cycles in different ulcer locations and stages.

**Figure 3:** Comparison of bleeding volume at different ulcer locations and stages.

**Figure 4:** Comparison of the bleeding of ulcer in different age groups within one year.

**Figure 5:** Comparison Chart of ulcer bleeding in different genders within one year.

**Table 1:** Location and stage of gastroduodenal ulcer bleeding within one year (data source: self-statistics of the study).

Ulcer location	Acute stage			Healing stage			Scar stage		
	Number of bleeding cases	Bleeding cycle	Bleeding volume	Number of bleeding cases	Bleeding cycle	Bleeding volume	Number of bleeding cases	Bleeding cycle	Bleeding volume
Cardia	11 (39.29)	32.6 ± 6.7	204 ± 65	6 (21.43)	183.8 ± 63.4	152 ± 43	9 (32.14)	104.7 ± 52.8	193 ± 57
Bottom	14 (40)	38.6 ± 6.3	126 ± 73	8 (22.86)	205.5 ± 74.2	122 ± 58	11 (31.43)	132.5 ± 57.4	139 ± 66
Big bend	22 (39.29)	41.2 ± 7.4	427 ± 126	14 (25)	172.4 ± 61.8	394 ± 135	18 (32.14)	116.2 ± 55.9	435 ± 138
Small bend	12 (38.71)	28.7 ± 5.4	513 ± 167	6 (19.35)	216.9 ± 65.2	536 ± 289	10 (32.26)	95.7 ± 49.8	589 ± 207
Sinus and angular notch	28 (37.33)	29.3 ± 6.4	1036 ± 283	17 (22.67)	194.0 ± 69.4	972 ± 401	21 (28)	121.6 ± 53.2	1152 ± 376
Pylorus	16 (37.21)	31.3 ± 6.1	624 ± 114	9 (20.93)	214.2 ± 73.6	690 ± 198	13 (30.23)	135.2 ± 58.5	668 ± 219
Duodenum	28 (38.36)	35.4 ± 6.6	1372 ± 389	19 (26.03)	228.6 ± 68.5	1152 ± 409	22 (30.14)	109.4 ± 51.2	1276 ± 384

**Table 2:** Comparison of bivariate *t*-test correlation based on staged observation data (data source: self-statistics of the study).

*t*		Acute stage			Healing stage			Scar stage		
*P*		Number of bleeding cases	Bleeding cycle	Bleeding volume	Number of bleeding cases	Bleeding cycle	Bleeding volume	Number of bleeding cases	Bleeding cycle	Bleeding volume
*Acute stage*	Number of bleeding cases	100								
		0.000								
	Bleeding cycle	—	100							
		—	0.000							
	Bleeding volume	—	—	100						
		—	—	0.000						

*Healing stage*	Number of bleeding cases	2.287	—	—	100					
		0.004	—	—	0.000					
	Bleeding cycle	—	3.298	—	—	100				
		—	0.006	—	—	0.000				
	Bleeding volume	—	—	4.383	—	—	100			
		—	—	0.004	—	—	0.000			

*Scar stage*	Number of bleeding cases	2.946	—	—	2.046	—	—	100		
		0.006	—	—	0.004	—	—	0.000		
	Bleeding cycle	—	2.943	—	—	2.511	—	—	100	
		—	0.074	—	—	0.006	—	—	0.000	
	Bleeding volume	—	—	3.273	—	—	2.438	—	—	100
		—	—	0.004	—	—	0.005	—	—	0.000

**Table 3:** Comparison of the correlation of *R*^2^ calibration of nonlinear curve estimation determination coefficient based on staged observation data (data source: self-statistics of the study).

*R* ^2^		Acute stage			Healing stage			Scar stage		
*P*		Number of bleeding cases	Bleeding cycle	Bleeding volume	Number of bleeding cases	Bleeding cycle	Bleeding volume	Number of bleeding cases	Bleeding cycle	Bleeding volume
*Acute stage*	Number of bleeding cases	—								
		—								
	Bleeding cycle	0.384	—							
		0.047	—							
	Bleeding volume	0.376	0.356	—						
		0.039	0.043	—						

*Healing stage*	Number of bleeding cases	0.367	0.322	0.335	—					
		0.042	0.038	0.037	—					
	Bleeding cycle	0.361	0.308	0.316	0.317	—				
		0.040	0.036	0.033	0.035	—				
	Bleeding volume	0.302	0.292	0.307	0.291	0.281	—			
		0.034	0.030	0.037	0.029	0.026	—			

*Scar stage*	Number of bleeding cases	0.294	0.281	0.283	0.276	0.266	0.257	—		
		0.031	0.029	0.032	0.025	0.024	0.023	—		
	Bleeding cycle	0.262	0.264	0.261	0.243	0.235	0.234	0.217	—	
		0.025	0.023	0.026	0.022	0.022	0.020	0.018	—	
	Bleeding volume	0.217	0.221	0.237	0.224	0.217	0.201	0.191	0.176	—
		0.021	0.022	0.020	0.019	0.020	0.016	0.015	0.011	—

**Table 4:** Comparison of bivariate *t*-test correlation based on observation data of ulcer location (data source: self-statistics of the study).

*t*	Cardia	Bottom	Big bend	Small bend	Sinus and angular notch	Pylorus	Duodenum
*P*							
*Cardia*	100						
	0.000						

*Bottom*	1.546	100					
	0.003	0.000					

*Big bend*	1.245	1.857	100				
	0.007	0.002	0.000				

*Small bend*	1.678	1.165	1.714	100			
	0.005	0.001	0.005	0.000			

*Sinus and angular notch*	1.167	1.547	2.087	2.204	100		
	0.006	0.004	0.005	0.004	0.000		

*Pylorus*	1.241	1.967	2.112	2.047	1.647	100	
	0.003	0.006	0.004	0.007	0.002	0.000	

*Duodenum*	1.015	2.647	2.107	2.309	2.005	1.921	100
	0.002	0.004	0.006	0.008	0.007	0.003	0.000

**Table 5:** Comparison of the correlation of R^2^ calibration of nonlinear curve estimation determination coefficient based on the observed data of ulcer location (data source: self-statistics of the study).

*R* ^2^	Cardia	Bottom	Big bend	Small bend	Sinus and angular notch	Pylorus	Duodenum
*P*							
Cardia	—						
	—						

Bottom	0.164	—					
	0.008	—					

Big bend	0.154	0.135	—				
	0.006	0.005	—				

Small bend	0.161	0.162	0.115	—			
	0.007	0.006	0.003	—			

Sinus and angular notch	0.137	0.153	0.132	0.114	—		
	0.005	0.005	0.006	0.002	—		

Pylorus	0.116	0.147	0.133	0.135	0.112	—	
	0.002	0.004	0.003	0.007	0.002	—	

Duodenum	0.167	0.162	0.127	0.189	0.106	0.215	—
	0.004	0.005	0.005	0.009	0.001	0.004	—

**Table 6:** Comparison of age and bleeding within one year (data source: self-statistics of the study).

		<30	30∼39	40∼50	>50
*Acute stage*	Number of bleeding cases	31 (19.87)	36 (23.08)	42 (26.92)	47 (30.13)
	Bleeding cycle	34.5 ± 5.8	39.4 ± 6.1	43.7 ± 5.4	46.3 ± 5.4
	Bleeding volume	539.5 ± 5.6	553.4 ± 6.2	578.3 ± 5.9	633.8 ± 6.2

*Healing stage*	Number of bleeding cases	13 (18.06)	17 (23.61)	20 (27.78)	22 (30.06)
	Bleeding cycle	233.4 ± 5.7	236.7 ± 5.3	240.6 ± 5.5	243.7 ± 5.2
	Bleeding volume	513.5 ± 6.2	534.1 ± 5.8	561.4 ± 6.4	598.7 ± 6.3

*Scar stage*	Number of bleeding cases	12 (17.14)	16 (22.86)	18 (25.71)	24 (34.29)
	Bleeding cycle	102.1 ± 4.5	142 ± 3.4	179.7 ± 5.1	201.2 ± 5.4
	Bleeding volume	642.1 ± 4.6	675.1 ± 4.8	690.4 ± 5.6	732.1 ± 5.1

**Table 7:** Comparison between gender and bleeding within one year (data source: self-statistics of the study).

		Male	Female
*Acute stage*	Number of bleeding cases	17(70.83)	7(29.17)
	Bleeding cycle	38.4 ± 4.8	31.5 ± 4.6
	Bleeding volume	523.3 ± 4.6	500.2 ± 4.8

*Healing stage*	Number of bleeding cases	15(78.95)	4(20.05)
	Bleeding cycle	245.7 ± 6.4	211.3 ± 5.4
	Bleeding volume	531.2 ± 4.4	498.4 ± 5.1

*Scar stage*	Number of bleeding cases	18(66.67)	9(33.33)
	Bleeding cycle	132.7 ± 5.6	101.7 ± 6.2
	Bleeding volume	627.8 ± 5.9	606.1 ± 5.2

## Data Availability

The data underlying the results presented in the study are available within the manuscript.
